RETRACTED

# Mechanical Performance Test and Numerical Simulation Analysis of Building Steel Plate and Concrete Composite Structure

**DOI:** 10.1155/2022/2156921

**Published:** 2022-07-20

**Authors:** Qian Liu

**Affiliations:** Anhui Vocational and Technical College, Hefei, 230063, Anhui, China

## Abstract

The study aims to continuously improve the level of the construction industry, such as the improvement of construction capacity and efficiency and reduction of the project cost and construction period, and find a specific way to improve the development of the construction industry. First, the study analyzes the research status of mechanical properties of horizontal joints, vertical joints, and the overall structure of worldwide prefabricated buildings. Next, the built-in steel fabricated concrete shear wall model is established. Moreover, the quasi-static experimental analysis is conducted on the joints of the fabricated shear wall with built-in section steel. The finite element software is used to analyze the numerical simulation test of the new built-in shear wall. According to the relevant test parameters, the finite element model is constructed, and the parameters are set. Finally, the shear wall model is established and tested by a simulation experiment, and the simulation results are compared with the numerical simulation results. The final results show that the proposed connection mode of the reinforced skeleton and new fabricated joints improves the stability of prefabricated buildings. The use of the quasi-static test to test the relevant performance parameters has a short calculation time, high efficiency, and high parameter optimization accuracy. It can better simulate the actual working conditions and the actual stress-strain and damage failure conditions. Moreover, the conclusion is drawn that the shear wall structure with steel plate concrete has good ductility and deformation capacity. The study has a certain reference significance for the construction optimization of steel plate concrete prefabricated buildings and related research in the future.

## 1. Introduction

New construction technology and its auxiliary means have been paid increasing attention by the engineering community with the vigorous development of new infrastructure in China. More advanced construction methods are needed because of the current requirements for environmental protection, the continuous reduction of the adult labor force in the construction industry, and the continuous rise in labor costs. The new built-in steel fabricated concrete building will become mainstream in the future. This building structure is of great significance in simplifying construction steps, improving construction quality, improving the management level, and reducing construction difficulty [1, 2].

RETRACTED

The current buildings are mainly reinforced concrete structures. The main advantages of concrete include good integrity, moldability, durability, fire resistance, and low project and maintenance costs. The concrete can be poured into an integral structure of various shapes and sizes. It can be prefabricated and cast-in-situ. Prefabrication is to make concrete components in the factory and then transport them to the construction site for assembly and connection to form a fabricated concrete structure. Cast-in-situ is to directly cast the concrete into the mold at the construction site to form an integral concrete structure. The definition of the prefabricated building is to convert the production of components and accessories in traditional construction methods into the factory in advance, transport them to the construction site in the construction process, and then assemble them on-site in the required position with safe and reliable connection [3]. After a period of development, the technology and equipment of prefabricated buildings have become mature. Traditional buildings are constructed directly on the construction site. However, for prefabricated buildings, the components are prefabricated in the factory and then transported to the construction site for assembly. Current prefabricated buildings are very popular in Japan, Europe, and America, but they are still in their infancy in China. According to the requirements of the Ministry of Housing and Urban-Rural Development of the People's Republic of China, by 2025, the proportion of prefabricated buildings in new buildings in China will be more than 50%.

With the continuous development of modern computer technology, the construction technology of engineering projects is also improving. The study expects to apply the emerging computer technology to the construction of prefabricated steel plate concrete structures. First, the research status of structural mechanical properties of worldwide prefabricated buildings is analyzed. Next, the model of built-in steel fabricated concrete shear wall is established. Moreover, the quasi-static experimental analysis of the joints of the fabricated shear wall with built-in section steel is carried out. The finite element software is used for numerical simulation and experimental analysis of the shear wall. Then, the finite element model is constructed, and the parameters are set according to the relevant test parameters. Finally, the shear wall model is established and tested by a simulation experiment. The experimental simulation results and numerical simulation results are analyzed. The final results show that using a quasi-static experiment to test the relevant performance parameters has a short calculation time, high efficiency, and high parameter optimization accuracy. The finite element analysis model used can better simulate the test conditions and simulate the stress, strain, displacement, damage process, and failure characteristics of prefabricated specimens. It is concluded that the steel plate concrete shear wall structure has good ductility and deformation capacity. The results have certain reference significance for building construction optimization and future research by using the assembly method under the development conditions of China's existing construction industry.

RETRACTED

## 2. Mechanical Property Experiment and Data Simulation Analysis

### 2.1. Research Status of Prefabricated Buildings

In the past two years, most industry insiders and the masses have recognized prefabricated buildings because of their multiple advantages. Assembly technology has also been widely used in the construction industry and has gradually become a new development trend. Prefabricated buildings rely more on professional hoisting teams to splice the components one by one through large mechanical equipment and hooks reserved on the components. It makes the construction process as convenient as building blocks.

The current situation of assembled buildings in the world is as follows: (1) single structure and shape. At present, the greatest difficulty of the prefabricated building is that the shape of the component structure is relatively single, and most are standardized components. The production of more complex components will significantly increase the construction cost and cannot achieve good economic benefits. (2) Production and transportation problems. In prefabricated buildings, since the components are directly transported to the site by the processing plant, the control of component quality is slightly insufficient. (3) The omission of embedded pipelines. At present, there are few qualified prefabricated building design units. Besides, the operation methods of many prefabricated buildings are not perfect. The omission of embedded pipelines is very common, seriously affecting the structure's safety [4, 5].

The current development status of prefabricated buildings in China is as follows: (1) with the increasing cost and insufficient standardization, the manufacturing price of prefabricated parts is consistently high, which makes the on-site installation process more troublesome than on-site pouring. (2) It is difficult to control the quality, and the test means of connection effect of various connection modes are cumbersome, which further increases the construction cost. Therefore, the shear wall has become the main stressed structure in prefabricated buildings, so its connection mode is the focus of research [6].

RETRACTED

#### 2.1.1. Shear Wall Horizontal Joint Structure

The stability of the shear wall with fabricated steel plate strip concrete is studied.  Figure 1 shows the horizontal joint structure of the shear wall.

The structure contains butted steel strips. Hence, it can effectively prevent the generation and development of cracks to improve the seismic energy dissipation capacity and ductility. The bolt in the structure can transfer the structure, stress, and its horizontal joint has a strong deformation ability. The research in recent years has successfully increased the performance of connectors. The horizontal joint structure in Figure 1(a) can greatly improve the seismic performance of the shear wall. Although the initial stiffness is slightly lower than that of the cast-in-situ type, its bearing performance is improved after the specimen is moved up [7, 8].

#### 2.1.2. Shear Wall Vertical Joint Structure

Figure 2 shows the vertical joint shear wall structure.

The failure form of the concrete wall in Figure 2 is bending shear failure. The failure process is divided into elastic failure, elastic-plastic failure, and softening failure. Compared with the cast-in-situ wall, there are macrovertical cracks in the internal joint of the shear wall in the quasi-static test. Therefore, it is determined that the brittle failure can be restrained, its deformation capacity is significantly increased, and its shear capacity is reduced considerably. The strength of the fabricated shear wall increases, while the ductility and energy dissipation capacity decrease. Therefore, for the quality and performance of the shear wall, the overall stress performance, bearing capacity, ductility, and rigidity of the vertical joint have been slightly enhanced, so it meets the stress standard of the wall [9].

#### 2.1.3. Integral Structure of the Shear Wall

Figure 3 shows the shear wall's overall internal structure and node structure.

Upper and lower horizontal cracks are the failure form of fabricated wallboard. After the plastic hinge forming, the microcrack is finally on the joint surface of the vertical connection, and the failure of the contact surface will significantly reduce the stiffness of the overall structure. A load of fabricated structure shear wall is similar to that of cast-in-situ, and the fundamental failure form and process are basically the same. The prefabricated parts of the assembly type have strong integrity, and the load on the joint is larger than that of the cast-in-place structure [10, 11].

RETRACTED

### 2.2. Quasi-Static Test of Shear Wall Joints

The geological movement where the house is located will cause the structure to vibrate back and forth in the horizontal direction, which can be simplified as the alternating action of the horizontal structure in the positive and negative directions. Because its duration is not long, it can be simplified as two alternating load movements in mutually perpendicular directions. Under the influence of the damping of the structure itself, the repetition times of the motion are not many, usually dozens of times. In special cases, the internal force, bending moment, shear force, and axial force of the structure will be carried out alternately due to the repeated action of load. Therefore, studying the prefabricated mixture embedded with structural steel is necessary. In addition to establishing the restoring force model, the hysteretic characteristics of shear wall components under repeated action are the basis of the whole process of analyzing the performance of structures and components.

#### 2.2.1. Experimental Methods and Objectives

The defects of the original concrete shear wall splicing method are analyzed, and a method is put forward. The universal beam is used to replace the restrained edge parts, embedded in the wall and welded with a steel structure to make the wall closely combined. The reason for choosing the universal beam is that it has a large cross-sectional area and is convenient for connection, making the connection of the upper and lower structures more convenient. The postcast layer in the connection area is fixed with a vertical steel bar to resist the horizontal slip trend [12]. The new fabricated shear wall is constructed.  Table 1 shows the experimental objectives of the study.

#### 2.2.2. Internal and External Structure Design of the Shear Wall

Figure 4 shows the zoning and numerical diagram of the shear wall's internal structure. The numerical unit is mm.

The universal beam is embedded in the core area of the shear wall, and a length more than the wall length is reserved in the up and down directions. However, the reserved length of the universal beam inside the wall is the same as the height of the connection area. Moreover, the connection of the walls at both ends is determined by welding the reserved universal beam. The universal beam is connected to the postcast layer between the two walls, and its height is 0.2 m. Stiffeners are added outside the flange to increase the bonding capacity between steel and concrete. In the two sections of walls, longitudinal and transverse stiffeners are added. The longitudinal distributed steel bars of the two sections of walls in the postcast layer must be anchored in the postcast layer. The transverse stiffener will pass through some universal beams to balance the stress distribution of the shear wall structure [13].  Table 2 shows the joint size and type.

RETRACTED

#### 2.2.3. Fabrication of Experimental Specimen

Formwork and support are made in the laboratory after processing and forming. Frame concrete is added, and wall structure and foundation pedestal construction are carried out first. After the completion of fabrication and 49 days of curing to make the concrete fully deformed, the pouring layer of concrete is poured [14].  Figure 5 shows the whole production flow chart.

Equation (1) is the calculation of the standard value *f*_*ck*_ of cube axial compressive strength. Equation (2) is the standard value of cube compressive strength *f*_*c*_. Equation (3) is the standard value of axial tensile strength *f*_*tk*_. Equation (4) is the calculation of concrete elastic modulus *E*. *f*_*cu*,*k*_ represents the standard value of cube compressive strength, and *α*_*c*1_ is the given coefficient.

(1) $$\begin{array}{c} f_{ck}=0.88\alpha_{c1}\alpha_{c1}f_{cu,k}, \end{array}$$

(2) $$\begin{array}{c} f_{c}=\frac{f_{ck}}{1.4}, \end{array}$$

(3) $$\begin{array}{c} f_{tk}=0.88\times 0.395f_{cu,k}^{0.55}{\left(1-1.645\delta \right)}^{0.45}, \end{array}$$

(4) $$\begin{array}{c} E=\frac{10^{5}}{2.2+\left(34.7/f_{cu,k}\right)}. \end{array}$$

### 2.3. Simulation Experiment

#### 2.3.1. Mechanical Property Test Items

The experiment aims to measure the horizontal load, displacement, and deformation of the shear wall under low cycle repeated horizontal load. In this way, the variation function relationship between load and other parameters, the strain relationship between steel bar and universal beam, and the deformation law of crack and specimen with time are obtained. The axial pressure is obtained by the Jack cooperating with the reaction frame, and the load is measured by the force sensor set on it. The actuator provides the repeated load. The automatic sensing device is used to obtain the experimental data information. The horizontal displacement value of the measured position is input and measured to study the stress-strain distribution law of the internal steel structure. Strain gauges are set up at a certain position of the specimen to measure stress and strain and collect data. The generation and propagation of cracks will be measured until the final complete failure of the wall.

#### 2.3.2. Selection and Erection of Stress and Strain Measuring Points

Before building the wall, a total of four steel structure resistance strain gauges shall be set at the pre- and postcast slab, respectively. Sixteen resistance strain gauges are placed on the steel structure, that is, universal beam and reinforcement. In addition, separate sensors are placed at each part of the bottom of the universal beam.

RETRACTED

#### 2.3.3. Load Loading of Specimen

The actuator is used to provide load. Mechanical tests and numerical simulations are conducted through the low-cycle repeated load provided. When carrying out load loading, it is necessary to make the vertical load stable, load at the top of the specimen, carry out vertical loading first, and then carry out transverse loading. Equation (5) shows the implementation of vertical load. Preloading is required before load loading. The complete load needs to be loaded to 40% of the total load first and then gradually loaded to 100% [15]. Equation (6) is the expression of the cracking load.

(5) $$\begin{array}{c} n=\frac{F}{f_{ck}A_{c}+f_{ak}A_{a}}, \end{array}$$

(6) $$\begin{array}{c} V=\left(\frac{F}{A}+f_{tk}\right)\frac{W}{H}, \end{array}$$

where *n* is the axial compression ratio, *F* is the axial pressure, *f*_*ck*_ represents the standard value of axial compressive strength, *f*_*ak*_ represents the standard value of the measured yield strength of universal beam, *A*_*c*_ represents the cross-sectional area of the shear wall, *A*_*a*_ refers to the cross-sectional area of the universal beam, *W* represents the work done by load, and *H* is the yield stress.

### 2.4. Finite Element Analysis

Abaqus is a set of powerful finite element software for engineering simulation, which can solve problems ranging from relatively simple linear analysis to many complex nonlinear problems.

#### 2.4.1. Establishment of Finite Element Model

Figure 6 displays the overall construction process of the finite element model.

#### 2.4.2. Setting of an Analysis Step

Abaqus is used for analysis. First, the parameters of the analysis step are set, and the maximum load steps are set to be slightly larger than the actual number of steps. The initial increment is set to 0.01, and an appropriate minimum increment value needs to be obtained through experiments.  Figure 7 shows the setting steps.

#### 2.4.3. Setting of Calculation Equation

Equations (8)–(12) are the calculation of concrete under uniaxial compression.

(7) $$\begin{array}{c} \sigma =\left(1-d_{c}\right)E_{c}\varepsilon , \end{array}$$

(8) $$\begin{array}{c} d_{t}=1-\frac{\rho_{c}n}{n-1+x^{n}},\;x\leq 1 \end{array}$$

(9) $$\begin{array}{c} x=\frac{\varepsilon }{\varepsilon_{c,r}}, \end{array}$$

(10) $$\begin{array}{c} \rho_{c}=\frac{f_{c,r}}{E_{c}\varepsilon_{c,r}}, \end{array}$$

(11) $$\begin{array}{c} n=\frac{E_{c}\varepsilon_{c,r}}{E_{c}\varepsilon_{c,r}-f_{c,r}}, \end{array}$$

where *a*_*c*_ represents the parameter value of the pressure stress-strain decreasing section, *f*_*c*,*r*_ represents the representative value of the compressive strength, *ε*_*c*,*r*_ is the compressive strain value corresponding to *f*_*c*,*r*_, *d*_*c*_ represents the compression damage evolution parameter, *σ* represents the compressive stress, *ε* represents the compressive strain, *E*_*c*_ represents deformation modulus, *ρ* represents compressive stress coefficient, *x* represents displacement, and *n* represents modulus coefficient. Equations (13)–(16) are the secondary loading stress of concrete.

(12) $$\begin{array}{c} \sigma =\left(\varepsilon -\varepsilon_{z}\right)E_{r}, \end{array}$$

(13) $$\begin{array}{c} E_{r}=\frac{\sigma_{un}}{\sigma_{un}-\sigma_{z}}, \end{array}$$

(14) $$\begin{array}{c} \varepsilon_{z}=\varepsilon_{un}-\left(\frac{\left(\varepsilon_{un}+\varepsilon_{ca}\right)\sigma_{un}}{\sigma_{un}+E_{c}\varepsilon_{ca}}\right)\frac{\varepsilon }{\varepsilon_{c,r}}, \end{array}$$

(15) $$\begin{array}{c} \varepsilon_{ca}=\text{max}\left(\frac{\varepsilon_{c}}{\varepsilon_{c}+\varepsilon_{un}},\frac{0.09\varepsilon_{un}}{\varepsilon_{c}}\right)\sqrt{\varepsilon_{c}u_{n},} \end{array}$$

where *ε*_*z*_ represents the residual strain when the load is unloaded to the zero stress point under compression; *E*_*r*_ represents the deformation modulus of secondary loading under compression; *σ*_*un*_ and *ε*_*un*_ represent the stress and strain at the beginning of unloading, respectively; *ε*_*ca*_ is the additional strain, and *ε*_*c*_ is the strain at the maximum stress under compression. The following equation shows the calculation of the concrete damage factor:

(16) $$\begin{array}{c} d_{k}=\frac{\left(1-\beta \right)\varepsilon^{in}E}{\alpha_{k}+\left(1-\beta \right)\varepsilon^{in}E}, \end{array}$$

where *d*_*k*_ represents the damage factor, *β* represents the proportional coefficient of plastic strain, and *ε*^*in*^ represents inelastic deformation. The following equation is the constitutive relationship expression of steel:

(17) $$\begin{array}{c} \sigma =E_{\varepsilon },\;\varepsilon <\varepsilon_{r}\\ \sigma =\sigma_{s}+E_{1}\left(\varepsilon -\varepsilon_{t}\right),\;\varepsilon \geq \varepsilon_{r}. \end{array}$$

where *σ* is the steel stress, *σ*_*s*_ represents the actual yield stress of steel, *ε*_*r*_ is the steel yield strain, *E*_1_ represents the slope of the straight line in the strengthened elastic-plastic curve, *E* represents the actual calculated value of elastic modulus, and *ε* is the strain just now.

RETRACTED

Displacement ductility is an important index to measure the elastic-plastic deformation capacity of the structure members. It refers to the ability of structure members to withstand deformation without significant reduction in bearing capacity. It can also be defined as the ability of structure members to withstand elastic-plastic deformation before final failure. Generally, the displacement ductility of structure members can be quantified by the displacement ductility coefficient [16].

## 3. Experimental and Numerical Simulation Results of Mechanical Properties

### 3.1. Skeleton Curve and Stiffness Change in the Mechanical Experiment

Figure 8 is the loading curve of the load of the test piece.

In Figure 8, S1 and S2 represent the skeleton curves of test pieces 1 and 2, respectively. Among them, the yield load of test piece 1 reaches 261.4 kN, and the yield displacement reaches 10.3 mm. The yield load of test piece 2 reaches 265 kN, and the yield displacement reaches 10.5 mm. It suggests that the ultimate strength will be higher and the maximum displacement will be smaller. When the limit displacement is reached, the displacement of test piece 2 will be smaller than that of test piece 1. The stiffness degradation curves of test pieces 1 and 2 will be closer and closer, and the stiffness change trend is slightly different during loading. Therefore, the stiffness of test pieces with large axial pressure will be larger, and the stiffness of the post pouring area will be greater than that of the foundation pedestal top.

### 3.2. Ductility Coefficient and Energy Dissipation Capacity

Table 3 is the comparison of the ductility coefficient of the test piece, and Figure 9 is the comparison diagram of energy dissipation capacity.

In Table 3, the ductility coefficient of the test piece exceeds 3, which means that the ductility is excellent. Therefore, it is proved that different axial compression ratios will have different effects on the ductility of the test piece and produce different ductility coefficients. After repeated loading, the energy consumed by the test piece can be calculated by the size of the closed block of the load-deformation curve. Due to the gradual increase of the displacement of the test piece, the energy dissipated will continue to increase, and the overall energy consumption and growth rate of the test piece with a relatively large axial compression ratio are large.

## 4. Conclusion

The study mainly optimizes the construction methods under the background of modern computer technology. First, the mechanical properties of horizontal joints, vertical joints, and overall structure of prefabricated buildings are analyzed. Then, the steel plate concrete prefabricated shear wall model is established. Moreover, the quasi-static experimental analysis of joints of steel plate concrete fabricated shear wall is carried out. The finite element software Abaqus is used to conduct numerical simulation and experimental analysis of the new fabricated shear wall. According to the relevant test parameters of the specimen obtained before, the finite element model is constructed, and the parameters are set. Finally, the shear wall model is established and tested by a simulation experiment. The experimental simulation results are compared with the numerical simulation results. Finally, it is proved that the proposed new joint connection method improves the stability of prefabricated buildings. Using a quasi-static test to test relevant performance parameters can better simulate the actual working conditions and simulate the actual stress-strain and damage failure. The shear wall structure of steel plate concrete has good ductility and deformation capacity and can correctly simulate the skeleton curve and the changing trend of stiffness.

RETRACTED

Although the study has achieved the expected research objectives and obtained valuable research conclusions, there are still multiple deficiencies in the research work. The following two factors limit the research conclusions. (1) Analysis of different building environments is insufficient. (2) Long-term construction data are not collected. They also point out the direction for future research, which will focus on the following two aspects: (1) simulation experiments on different building environments will be conducted to judge mechanical properties and (2) the scale of the data set will be further expanded, the number of training will be increased, and a more detailed numerical simulation will be used to analyze it.

## Figures and Tables

**Figure 1:** Shear wall horizontal joint structure: (a) shear wall of steel plate strip concrete and (b) prefabricated shear wall with reserved postcast area at the bottom.

**Figure 2:** Vertical joint shear wall structure: (a) embedded position in steel plate bolt wall and (b) structure in fabricated shear wall.

**Figure 3:** Shear wall structure: (a) fabricated shear wall integral structure and (b) shear wall joint.

**Figure 4:** Internal structure of shear wall: (a) partition diagram of shear wall structure and (b) dimension diagram of shear wall joint.

**Figure 5:** Production flow chart of the test piece.

**Figure 6:** Overall construction process of finite element model.

**Figure 7:** Setting of numerical simulation analysis steps.

**Figure 8:** Load curve of the test piece: (a) skeleton curve of the test piece and (b) stiffness change of test pieces 1 and 2 during positive and negative loading of the test piece.

RETRACTED

**Figure 9:** Comparison of energy dissipation capacity.

**Table 1:** Experimental objectives of the study.

Serial number	Specific description
1	The failure process and main failure modes of shear wall joints are analyzed.
2	The seismic performance of shear wall joints with different axial compression ratios is compared and analyzed.
3	The load and displacement results of cracking, yield, limit, and other stages are collected through the quasi-static test of joints.
4	The restoring force curve model of the shear wall is made, and the model's effectiveness is verified.
5	The performance parameters obtained from the experiment are collected as the basis of finite element analysis.

**Table 2:** Joint size and type.

Serial number	Name	Size and installation position
1	Lower foundation pedestal of shear wall	500 mm^*∗*^1,900 mm^*∗*^500 mm; it is anchored in the reserved hole of the floor with bolt columns.
2	Horizontally and vertically distributed steel bars and stirrups arranged around the section steel in the core area of the wall	HPB300 steel bar with a diameter of 6.5 mm is selected, and the transverse distribution steel bar is 2^*∗*^ɸ 6.5 mm^*∗*^200 mm. The upper 300 mm of the shear wall is the loading area; the horizontal distribution steel bar spacing is 100 mm; and the vertical distribution steel bar is 10ɸ 6.5 mm.
3	Wall concrete	Cast-in-situ concrete of C50. No. 10 universal beam (100 mm^*∗*^68 mm^*∗*^4.5 mm^*∗*^7.6 mm) shall be used in the wall restraint area, but welds shall be used for connection, and the weld strength shall not be lower than that of the base metal.
4	Foundation pedestal	C50 concrete, HRB400 steel bar with a diameter of 18 mm.

**Table 3:** Comparison of ductility coefficient of the test piece.

Test piece	Limit displacement (mm)	Yield displacement (mm)	Ductility coefficient (mm)
S1	36.9	9.32	4.12
S2	35.1	10.6	3.31

## Data Availability

The data used to support the findings of this study are available from the author upon request.
